RETRACTED

# Excessive mitochondrial fragmentation triggered by erlotinib promotes pancreatic cancer PANC-1 cell apoptosis via activating the mROS-HtrA2/Omi pathways

**DOI:** 10.1186/s12935-018-0665-1

**Published:** 2018-10-22

**Authors:** Jun Wan, Jie Cui, Lei Wang, Kunpeng Wu, Xiaoping Hong, Yulin Zou, Shuang Zhao, Hong Ke

**Affiliations:** 1 Department of Pharmacy, Third Clinical Medical College, Three Gorges University, Gezhouba Group Central Hospital, Yichang, 443002 Hubei China; 2 Department of Pathogenic Biology, School of Medicine, China Three Gorges University, Yichang, 443002 Hubei China; 3 Department of Oncology, Third Clinical Medical College, Three Gorges University, Gezhouba Group Central Hospital, No. 60 Qiaohu Lake Road, Xiling District, Yichang, 443002 Hubei China

**Keywords:** Erlotinib, Mitochondrial fragmentation, Mitochondrial apoptosis, mROS, HtrA2/Omi

## Abstract

**Background:**

Mitochondrial fragmentation drastically regulates the viability of pancreatic cancer through a poorly understood mechanism. The present study used erlotinib to activate mitochondrial fragmentation and then investigated the downstream events that occurred in response to mitochondrial fragmentation.

**Methods:**

Cell viability and apoptosis were determined via MTT assay, TUNEL staining and ELISA. Mitochondrial fragmentation was measured via an immunofluorescence assay and qPCR. siRNA transfection and pathway blockers were used to perform the loss-of-function assays.

**Results:**

The results of our study demonstrated that erlotinib treatment mediated cell apoptosis in the PANC-1 pancreatic cancer cell line via evoking mitochondrial fragmentation. Mechanistically, erlotinib application increased mitochondrial fission and reduced mitochondrial fusion, triggering mitochondrial fragmentation. Subsequently, mitochondrial fragmentation caused the overproduction of mitochondrial ROS (mROS). Interestingly, excessive mROS induced cardiolipin oxidation and mPTP opening, finally facilitating HtrA2/Omi liberation from the mitochondria into the cytoplasm, where HtrA2/Omi activated caspase-9-dependent cell apoptosis. Notably, neutralization of mROS or knockdown of HtrA2/Omi attenuated erlotinib-mediated mitochondrial fragmentation and favored cancer cell survival.

**Conclusions:**

Together, our results identified the mROS-HtrA2/Omi axis as a novel signaling pathway that is activated by mitochondrial fragmentation and that promotes PANC-1 pancreatic cancer cell mitochondrial apoptosis in the presence of erlotinib.

**Electronic supplementary material:**

The online version of this article (10.1186/s12935-018-0665-1) contains supplementary material, which is available to authorized users.

RETRACTED

## Background

Pancreatic cancer is the fourth leading cause of cancer-related death worldwide [1]. Although the incidence of pancreatic cancer is relatively low, approximately 3.2% of all new cancer cases in the United States, the 5-year survival rate is 8.5% in patients diagnosed with pancreatic cancer. In addition, the detection rate of early pancreatic cancer remains low due to the lack of specific symptoms. Accordingly, most patients (52%) are diagnosed with distant metastasis [2], and, unfortunately, the 5-year relative survival of patients with metastatic pancreatic cancer is less than 2% [3]. Although smoking and health history can affect the risk of pancreatic cancer, the pathogenesis of pancreatic cancer development is not completely understood. Therefore, exploring the molecular features of pancreatic cancer growth and death is vital to control the disease progression and bring more clinical benefits to patients with pancreatic cancer.

The biological behavior of cancer is closely regulated by mitochondria [4, 5]. Sufficient ATP supply, intracellular calcium homeostasis, metabolic signaling transduction, and cell apoptosis management are affected by mitochondria [6–8]. In addition, mitochondria are also the key target of several chemotherapeutics and radiotherapies [9]. A recent study has reported that pancreatic cancer death, proliferation and metastasis are modulated by mitochondrial homeostasis, especially mitochondrial fission [10]. Excessive mitochondrial fission induces cancer cell oxidative injury and subsequently mediates mitochondrial ATP depletion; this effect impairs PANC-1 cell proliferation and evokes mitochondrial apoptosis [10]. Notably, this conclusion is also supported by other studies. In colorectal cancer, the activation of mitochondrial fission is associated with SW837 cell apoptosis and migration inhibition [11]. In gastric cancer, abnormal mitochondrial fission contributes to cancer cell oxidative stress and energy undersupply [12]. In breast cancer, Drp1-mediated mitochondrial fission suppresses breast cancer cell invasion [13]. This information indicates that mitochondrial fission has a well-characterized role in the regulation of cancer viability. However, the downstream molecular events of mitochondrial fission activation remain to be discovered.

Based on a previous study in a mouse model of cardiac ischemia reperfusion injury, the activation of mitochondrial fission promotes the formation of mitochondrial fragmentation, and these mitochondrial debris contain a decreased mitochondrial potential [14]. In addition, mitochondrial fragmentation can activate cell death via two mechanisms [15]; one mechanism is driven via HK2/VDAC1 disassociation-mediated mPTP opening, and the other involves mROS-induced cardiolipin oxidation. Notably, mitochondrial ROS (mROS) overloading, as a primary result of mitochondrial fragmentation [16], has been noted in different disease models such as those of gastric cancer [17], breast cancer [18], and leukemia [19]. Subsequently, excessive mitochondrial oxidative injury can activate the HtrA2/Omi-related apoptotic pathway in a manner that is dependent on caspase-9 activity [11]. This evidence indicates that the downstream effectors of mitochondrial fragmentation include mROS overproduction, HtrA2/Omi upregulation, caspase-9 activation and mitochondrial apoptosis augmentation. Given these factors, we want to know whether mitochondrial fragmentation regulates pancreatic cancer viability via mROS-HtrA2/Omi-caspase-9 pathways.

RETRACTED

To this end, erlotinib is the first-line anti-tumor drug for the treatment of pancreatic cancer in the clinic [20]. Several human studies have verified the efficacy of erlotinib in improving the 5-year survival rate of patients with pancreatic cancer [21, 22]. Molecular investigations report that several biological processes are modulated by erlotinib, including mTOR inhibition [23], epidermal growth factor receptor downregulation [24], and epidermal interstitial transformation (EMT) suppression [25]. However, no study that explores the role of erlotinib in triggering mitochondrial stress has been conducted. In the present study, erlotinib was applied to activate mitochondrial fragmentation in a human PANC-1 pancreatic cancer cell line. Then, we explored the regulatory mechanism of mitochondrial fragmentation on cell viability in the presence of erlotinib.

## Methods and materials

### Pancreatic carcinoma cell lines

The PANC-1 (ATCC^®^ CRL-1469™) and MIA PaCa-2 (ATCC^®^ CRL-1420™) pancreatic cell lines were used in the present study. These cells were cultured in Dulbecco’s modified Eagle’s medium (DMEM) (Thermo Fisher Scientific, Waltham, MA) supplemented with 10% fetal bovine serum (FBS) (Thermo Fisher Scientific, Waltham, MA) at 37 °C in a 5% CO_2_ atmosphere. Different doses of erlotinib (ERL, Sigma. Cat. No. SML2156) were incubated with the cancer cells for 24 h, and these concentrations of ERL were chosen according to a previous study [26]. FCCP (5 μm, Selleck Chemicals, Houston, TX, USA) and mitochondrial division inhibitor 1 (Mdivi1; 10 mM; Sigma-Aldrich; Merck KGaA) were used to activate and inhibit mitochondrial fragmentation, respectively, according to a previous study. To repress mROS overproduction, mitochondrial-targeted antioxidant MitoQ (2 μM, MedKoo Biosciences, Inc.; CAT#: 317102) was used.

RETRACTED

### Western blotting and antibodies

Cells were scraped in RIPA lysis buffer (Beyotime, Shenzhen, Guangdong, China). The lysates (50–70 µg) were separated by 10% SDS-polyacrylamide gel (10–15%) electrophoresis (SDS-PAGE). Proteins were electrotransferred onto the Pure Nitrocellulose Blotting membrane (Life Sciences) (Millipore, Bedford, MA, USA) and then blocked with 5% nonfat milk for 2 h at room temperature [27]. After washing with TBST three times, the membranes were incubated at 4 °C overnight with the following primary antibodies: HrtA2/Omi (:1000; Abcam; #ab32092), caspase9 (1:1000, Cell Signaling Technology, #9504), Bax (1:1000, Cell Signaling Technology, #2772), Opa1 (1:1000, Abcam, #ab42364), Mfn2 (1:1000, Abcam, #ab56889), Tom20 (1:1000, Abcam, #ab186735), CDK4 (1:1000, Abcam, #ab137675), Cyclin D1 (1:1000, Abcam, #ab134175), Bcl2 (1:1000, Cell Signaling Technology, #3498), Bad (:1000; Abcam; #ab90435), survivin (1:1000, Cell Signaling Technology, #2808), cyt-c (1:1000; Abcam; #ab90529), complex III subunit core (CIII-core2, 1:1000, Invitrogen, #459220), complex II (CII-30, 1:1000, Abcam, #ab110410), complex IV subunit II (CIV-II, 1:1000, Abcam, #ab110268). Next, the membranes were visualized using an enhanced chemiluminescence system (ECL; Pierce Company, USA) [28].

### MTT assay, caspase activity detection and LDH release assay

MTT was used to analyze the cellular viability [29]. Cells (1 × 10^6^ cells/well) were cultured on a 96-well plate at 37 °C with 5% CO_2_. Then, 40 µl of MTT solution (2 mg/ml; Sigma-Aldrich) was added to the medium for 4 h at 37 °C with 5% CO_2_. Subsequently, the cell medium was discarded, and 80 µl of DMSO was added to the wells for 1 h at 37 °C with 5% CO_2_ in the dark. The OD of each well was observed at A490 nm via a spectrophotometer (Epoch 2; BioTek Instruments, Inc., Winooski, VT, USA). To analyze changes in caspase-9, caspase-9 activity kits (Beyotime Institute of Biotechnology, China; Catalog No. C1158) were used according to the manufacturer’s protocol [30]. In brief, to measure caspase-9 activity, 5 μl of LEHD-p-NA substrate (4 mM, 200 μM final concentration) was added to the samples for 1 h at 37 °C. Then, the absorbance at 400 nm was recorded via a microplate reader to reflect the caspase-3 and caspase-9 activities. To analyze caspase-3 activity, 5 μl of DEVD-p-NA substrate (4 mM, 200 μM final concentration) was added to the samples for 2 h at 37 °C [31].

### ELISA

Glutathione (GSH, Thermo Fisher Scientific Inc., Waltham, MA, USA; Catalog No. T10095), glutathione peroxidase GPX, (Beyotime Institute of Biotechnology, China; Catalog No. S0056) and SOD (Thermo Fisher Scientific Inc., Waltham, MA, USA; Catalog No. BMS222TEN) were measured according to the manufacturer’s instructions using a microplate reader (Epoch 2; BioTek Instruments, Inc.) [32]. Cellular ATP generation was measured to reflect mitochondrial function. Firstly, cells were washed three times with cold PBS at room temperature. Subsequently, a luciferase-based ATP assay kit (CellTiter-Glo^®^ Luminescent Cell Viability Assay; cat. no. G7570; Promega Corporation, Madison, WI, USA) was used to analyze ATP content, according to the manufacturer’s protocols. ATP production was measured using a microplate reader at the wavelength of 570 nm (Epoch 2; BioTek Instruments, Inc., Winooski, VT, USA) [33].

RETRACTED

### Immunostaining

Cells were washed twice with PBS, permeabilized in 0.1% Triton X-100 overnight at 4 °C. After the fixation procedure, the sections were cryoprotected in a PBS solution supplemented with 0.9 mol/l of sucrose overnight at 4 °C [34]. The primary antibodies used in the present study were as follows: caspase9 (1:1000, Cell Signaling Technology, #9504), Mff (1:1000, Cell Signaling Technology, #86668), Tom20 (1:1000, Abcam, #ab186735), HrtA2/Omi (1:1000; Abcam; #ab32092).

### Small interfering RNA transfection

To inhibit HtrA2/Omi expression, two independent siRNAs against HtrA2/Omi were transfected into PANC-1 cells according to a previous study [27]. Briefly, the cells were seeded onto 6-well plates and then incubated with Opti-Minimal Essential Medium (Invitrogen; Thermo Fisher Scientific, Inc.) for 24 h. Then, Lipofectamine^®^ 2000 transfection reagent (Thermo Fisher Scientific, Inc.) was added into the medium of PANC-1 cells and supplemented with 5 nmol/l siRNA solution. Transfection was performed for 48 h, and then the cells were collected. Western blotting was used to verify the transfection efficiency.

### Detection of mitochondrial membrane potential and mPTP opening

To observe the mitochondrial potential, JC-1 staining (Thermo Fisher Scientific Inc., Waltham, MA, USA; Catalog No. M34152) was used. Then, 10 mg/ml JC-1 was added to the medium for 10 min at 37 °C in the dark to label the mitochondria. Normal mitochondrial potential showed red fluorescence, and damaged mitochondrial potential showed green fluorescence [35]. The mPTP opening rate was detected using calcein-AM (Sigma, Cat. No. 17783) as described previously [36]. Briefly, cells were incubated with calcein-AM for 30 min at 37 °C in the dark. Next, PBS was used to wash the cells three times. Finally, the optical density (OD) at an absorbance of 579 nm was recorded using a multifunction microplate reader (Epoch 2; BioTek Instruments, Inc., Winooski, VT, USA). The mPTP opening rate was calculated as a ratio to that of the control group [14]. The relative mPTP opening was measured as a ratio to that of the control group.

RETRACTED

### TUNEL assay and cardiolipin staining

Apoptotic cells were detected with an In Situ Cell Death Detection Kit (Thermo Fisher Scientific Inc., Waltham, MA, USA; Catalog No. C1024) according to the manufacturer’s protocol. Briefly, cells were fixed with 4% paraformaldehyde at 37 °C for 15 min. Blocking buffer (3% H_2_O_2_ in CH_3_OH) was added to the wells, and then cells were permeabilized with 0.1% Triton X-100 in 0.1% sodium citrate for 2 min on ice. The cells were incubated with TUNEL reaction mixture for 1 h at 37 °C. DAPI (Sigma-Aldrich, St. Louis, MO, USA) was used to counterstain the nuclei, and the numbers of TUNEL-positive cells were recorded [37]. Cardiolipin oxidation was stained with 10-*N*-nonylacridine orange (NAO; 2 mmol/l; Molecular Probes, Eugene, OR, USA). Under normal conditions, NAO interacts with nonoxidized cardiolipin and generates a characteristic green fluorescence. However, upon cardiolipin oxidation, NAO cannot interact with cardiolipin, and this result is accompanied by a drop in green fluorescence. Accordingly, the green fluorescence intensity of NAO was used to quantify the cardiolipin oxidation with the help of Image-Pro Plus 6.0; Media Cybernetics, Rockville, MD, USA) [16].

### RNA extraction and qPCR analysis

For mRNA expression analysis, total RNA was isolated using Trizol (Invitrogen, Carlsbad, California, USA) according to a previous study. Then, cDNA was synthesized using 1 mg RNA and the First-Strand Synthesis Kit (Fermentas, Flamborough, Ontario, Canada) according to a previous study [38]. The cycling conditions were as follows: 92 °C for 7 min, 40 cycles of 95 °C for 20 s and 70 °C for 45 s. β-actin was amplified as an internal standard. All the primer sequences are listed below: Drp1 (forward prime 5′-CATGGACGAGCTGGCCTTC-3′, reverse prime 5′-ATCCTGTAGTGATGTATCAGG-3′), Mff (forward prime 5′-TGTCCAGTCCGTAACTGAC-3′, reverse prime 5′-TTCGATACCTGACTTAC-3′), Mfn2 (forward prime 5′-CCTCTTGATCCTGATCTTAACGT-3′, reverse prime 5′-GGACTACCTGATTGTCATTC-3′), OPA1 (forward prime 5′-GCTACTTGTGAGGTCGATTC-3′, reverse prime 5′-GCCGTATACCGTGGTATGTCTG-3′) [14].

### EdU staining

EdU staining was performed to analyze the cell proliferation according to a previous study [39]. The EdU incorporation assay was performed using the EdU kit (cat. no. A10044; Thermo Fisher Scientific Inc.). Briefly, EdU (2 nM/well) was diluted in complete culture medium, and the cells were incubated with the dilution for 2 h at 37 °C. Subsequently, the cells were fixed with 4% paraformaldehyde for 15 min at 37 °C and were incubated with Apollo Staining reaction liquid for 30 min. DAPI was used to counterstain the nuclei for 15 min at room temperature under a digital microscope system (IX81; Olympus Corporation).

RETRACTED

### Flow cytometry assay

Flow cytometry was applied as a quantitative method for evaluating mitochondrial ROS levels according to a previous study [4]. In brief, PANC-1 cells were seeded onto 6-well plates and then treated with erlotinib. Subsequently, the cells were isolated using 0.25% trypsin and then incubated with MitoSOX red mitochondrial superoxide indicator (Molecular Probes, USA) for 30 min in the dark at 37 °C. Subsequently, PBS was used to wash cell two times, and then the cells were analyzed with a FACS Calibur Flow cytometer. Data were analyzed by FACS Diva software. The experiment was repeated three times to improve the accuracy [39]. The number of apoptotic cells was analyzed quantitatively using the Annexin V–FITC/PI Apoptosis Detection Kit (BD Biosciences, USA). Aſter treatment, the cells were harvested, resuspended in 200 µl of binding buffer, and then incubated with 5 µl of Annexin V–FITC/binding buffer mixture (30 min, 37 °C) in the dark. Subsequently, the cells were incubated with 10 µl of propidium iodide for 5 min and immediately analyzed by bivariate flow cytometry using a BD FACSCalibur cytometer [36].

### Statistical analysis

Data are expressed as the mean ± SE of triplicate samples. Statistical analysis for multiple comparisons was analyzed by a one-way analysis of variance (ANOVA) followed by Bonferroni’s multiple comparison test. p values below 0.05 were considered statistically significant.

## Results

### Erlotinib dose-dependently promotes PANC-1 pancreatic cancer cell apoptosis

First, erlotinib was incubated with PANC-1 pancreatic cancer cells. Then, cell viability was observed using the MTT assay and LDH-cytotoxicity assay. Compared to the control group, erlotinib treatment reduced the viability of PANC-1 cells (Fig. 1a, b), and this effect was achieved in a dose-dependent manner. This finding was also found in erlotinib-treated PaCa-2 pancreatic cancer cells (Fig. 1c, d). To explore whether the reduction in cell viability was attributable to excessive cell apoptosis, the TUNEL assay was used. The number of TUNEL-positive cells was counted as the apoptotic index. As shown in Fig. 1e, f, erlotinib dose-dependently increased the apoptotic index in PANC-1 cells. Similarly, the number of TUNEL-positive cells was also elevated in PaCa-2 cells upon exposure to erlotinib (Fig. 1e, g). Furthermore, since cell apoptosis is primarily executed via caspase-3 activation, caspase-3 activity was determined via ELISA. Compared to the control group, caspase-3 activity was relatively increased in response to erlotinib treatment (Fig. 1h), which is suggestive of caspase-3 activation by erlotinib. This alteration was also noted in PaCa-2 cells (Fig. 1I). These data were further supported via quantitative analysis of cell apoptosis with the help of flow cytometry (Additional file 1: Figure S1). Together, our results indicated that erlotinib dose-dependently promoted PANC-1 and PaCa-2 cell apoptosis. Notably, no phenotypic difference was noted in erlotinib-mediated apoptosis in PANC-1 cells or PaCa2 cells, and thus PANC-1 cells were used in the following study. In addition, we have found that the minimum concentration of erlotinib that induces cell death was 10 μM, and thus, 10 μM erlotinib was used to conduct the molecular investigations.

RETRACTED

**Fig. 1:** Erlotinib promotes PANC-1 apoptosis in a concentration-dependent fashion. **a** The MTT assay for PANC-1 viability. Different doses of erlotinib were added to the medium of PANC-1 cells. **b** LDH release was used to evaluate the cell death in PANC-1 cells in the presence of erlotinib. **c** The MTT assay for PaCa-2 cells in the presence of erlotinib treatment. **d** LDH release was used to evaluate the cell death in PaCa-2 cells in the presence of erlotinib. **e** TUNEL staining for apoptotic PANC-1 cells and PaCa-2 cells. The number of TUNEL-positive cells was recorded. **f** Quantification of the TUNEL assay in PANC-1 cells. **g** The TUNEL assay for PaCa-2 cells in response to erlotinib treatment. The percentage of TUNEL-positive PaCa-2 cells was recorded. **h**, **i** Caspase-3 activity was determined using an ELISA in PANC-1 cells and PaCa-2 cells. ^#^*p *< 0.05 vs. control group

### Erlotinib induces mitochondrial fragmentation in PANC-1 pancreatic cancer cells via elevating mitochondrial fission and repressing mitochondrial fusion

Subsequently, the mitochondrial morphology was observed via an immunofluorescence assay using a Tom-20 antibody [40]. Compared to the control group, we found that erlotinib treatment mediated the formation of mitochondrial fragmentation (Fig. 2a). Then, the average length of the mitochondria was measured after erlotinib treatment and was used to quantify mitochondrial fragmentation. As shown in Fig. 2b, the mean length of the mitochondria was ~ 9.1 μm at baseline. However, after treatment with erlotinib, the mean length of mitochondria was reduced to ~ 2.3 μm (Fig. 2b). In addition, the fluorescence intensity of Mff, an activator of mitochondrial fragmentation, was obviously increased in response to erlotinib treatment compared to that in control group (Fig. 2c). Subsequently, to further confirm the promotive effect of erlotinib on mitochondrial fragmentation, Mdivi-1, an antagonist of mitochondrial fragmentation, was added into the medium of erlotinib-treated cells. Meanwhile, FCCP, an agonist of mitochondrial fragmentation, was used to incubate with normal cells, which was used as the positive control group. Then, mitochondrial fission, mitochondrial length and Mff expression were evaluated again. Compared to the control group, FCCP triggered mitochondrial fragmentation and upregulated Mff expression, similar to the results obtained via supplementation with erlotinib (Fig. 2a–c). However, Mdivi-1 treatment abrogated the promotive effect of erlotinib on mitochondrial fragmentation.

RETRACTED

**Fig. 2:** Erlotinib activates mitochondrial fragmentation in PANC-1 cells. **a** Mitochondrial fragmentation was determined using an immunofluorescence assay. Tom-20 was used to stain the mitochondria, and the average length of the mitochondria was calculated to quantify mitochondrial fragmentation. Mff antibody was used to lable the Mff, an mitochondrial fragmentation activator. FCCP and Mdivi-1 were used to activate or inhibit mitochondrial fragmentation, respectively. **b** Quantification of the mitochondrial length. **c** The relative Mff fluorescence intensity was evaluated in the presence of erlotinib treatment. FCCP and Mdivi-1 was used to activate or inhibit mitochondrial fragmentation, respectively. Mdivi-1, an antagonist of mitochondrial fragmentation, was added into the medium of erlotinib-treated cells. Meanwhile, FCCP, an agonist of mitochondrial fragmentation, was used to incubate with normal cells, which was used as the positive control group. **d**–**g** The alterations of mitochondrial fission/fusion-related factors were measured using qPCR. Drp1 and Mff were pro-fission proteins, and their expressions were significantly increased in response to erlotinib treatment. In contrast, Mfn2 and Opa1 were pro-fusion factors, and their levels were downregulated by erlotinib application. **h–j** Western blotting for Mfn2 and Opa1 in response to erlotinib treatment. *p < 0.05

Notably, the fragmented mitochondria could be the result of increased mitochondrial fission and decreased mitochondrial fusion. To verify the alterations of mitochondrial fission/fusion, qPCR was performed to analyze the transcription factors that are related to mitochondrial fission/fusion. In response to erlotinib treatment, the transcription of pro-fission factors such as Drp1 and Mff were significantly upregulated (Fig. 2d–g), indicative of mitochondrial fission activation by erlotinib. In contrast, the transcription and expression of pro-fusion factors, such as Mfn2 and Opa1 were obviously downregulated in response to erlotinib treatment (Fig. 2d–j), suggesting that mitochondrial fusion was repressed by erlotinib. Together, our results confirmed that erlotinib promoted mitochondrial fragmentation in PANC-1 cells.

RETRACTED

### Mitochondrial fragmentation induces oxidative stress via mitochondrial ROS (mROS)

Additional experiments were performed to explore the downstream events of mitochondrial fragmentation. Based on a previous study, mitochondrial fragmentation was associated with cellular oxidative stress via mROS overloading [41]. To confirm this, a mROS probe and flow cytometry were used to quantify mROS levels after erlotinib treatment. As shown in Fig. 3a, b, the level of mROS was significantly elevated in response to erlotinib treatment. To validate whether mitochondrial fragmentation was required for mROS overloading, Mdivi-1 and FCCP were used. FCCP treatment elevated the ROS production in control group, similar to the results obtained vis supplementation of erlotinib, However, Mdivi-1 application attenuated erlotinib-mediated mROS overloading (Fig. 3a, b), indicating the necessary role that is played by mitochondrial fragmentation in mROS generation. Excessive mROS production would induce cellular oxidative injury. To confirm this, an ELISA assay was used to observe alterations in the levels of cellular antioxidants. Compared to the control group, the concentration of Mn-SOD, GSH and GPX were markedly reduced after erlotinib treatment (Fig. 3c–e). In contrast, the level of MDA, an end product of the peroxidation of lipids in the cell membrane, was increased in response to erlotinib treatment (Fig. 3f). Interestingly, blockade of mitochondrial fragmentation via Mdivi-1 could decrease the level of antioxidants and suppress the production of MDA (Fig. 3c–f). Excessive oxidative injury can also disrupt cellular energy metabolism. Accordingly, total ATP production was measured using ELISA. Compared to the control group, erlotinib treatment significantly reduced the ATP production in PANC-1 cells (Fig. 3g), and this effect could be reversed by Mdivi-1. Furthermore, we also found that the expression of proteins related to mitochondrial ATP synthesis were notably downregulated in response to erlotinib (Fig. 3h–k); this effect was abrogated by Mdivi-1. Accordingly, our data indicated that mitochondrial fragmentation evoked mitochondrial ROS overloading and oxidative stress in PANC-1 cells.

**Fig. 3:** Mitochondrial fragmentation promotes mitochondrial ROS (mROS) overproduction. **a** The levels of mROS was measured using a mitochondrial ROS probe, and a quantitative analysis of mROS was conducted using flow cytometry. **b** Quantification of mROS in PANC-1 cells treated with erlotinib. The antagonist Mdivi-1 was added to the medium of PANC-1 cells to inhibit the activity of mitochondrial fragmentation. **c**–**f** An ELISA was used to evaluate the concentrations of factors involved in the cellular redox status. Mn-SOD, GSH and GPX are antioxidant factors whereas MDA is an end product of cellular membrane oxidation, was detected using an ELISA kit. **g** PANC-1 cells were treated with erlotinib or Mdivi-1, and then cellular total ATP production was measured using an ELISA. **h**–**k** Mitochondrial respiratory complex expression was determined by western blotting in the presence of erlotinib. *p < 0.05

RETRACTED

### Mitochondrial fragmentation-mediated mROS promotes HtrA2/Omi liberation

Next, experiments were performed to observe the consequence of mROS-mediated cell oxidative stress. Based on a previous report [42], excessive mROS could cause mitochondrial membrane permeabilization, which facilitates the translocation of mitochondrial proapoptotic factors to the nucleus/cytoplasm [43]. In the present study, an immunofluorescence analysis demonstrated that erlotinib increased the migration of HtrA2/Omi to nucleus when compared to the control group (Fig. 4a, b). Interestingly, this effect of erlotinib could be abolished via Mdivi-1 (Fig. 4a, b). Subsequently, western blotting was performed to quantify HtrA2/Omi liberation. As shown in Fig. 4c–e, compared to the control group, erlotinib treatment increaased the levels of cytoplasmic HtrA2/Omi (cyto-Htra2/Omi) and reduced the expression of mitochondrial HtrA2/Omi (mito-HtrA2/Omi). Similar results were also observed in cytochrome c (cyt c) liberation from mitochondria into cytoplasm (Fig. 4c–f). However, Mdivi-1 treatment repressed the erlotinib-mediated HtrA2/Omi and cyt c translocation from mitochondria into the cytoplasm. These results indicated that mitochondrial fragmentation accounted for HtrA2/Omi liberation.

**Fig. 4:** Mitochondrial fragmentation-mediated mROS induces HtrA2/Omi liberation. **a**, **b** Immunofluorescence measurements of HtrA2/Omi in response to erlotinib treatment. Mdivi-1 was used to inhibit mitochondrial fragmentation. **c**–**f** Cytoplasmic HtrA2/Omi (cyto-HrA2/Omi), cytoplasmic cyt c (cyto-cyt c), mitochondrial HtrA2/Omi (mito-HtrA2/Omi) and mitochondrial cyt c (mito-cyt c) were determined using western blotting analysis. **g**, **h** Cardiolipin oxidation was observed using an NAO probe. In response to cardiolipin oxidation, NAO could not bind to oxidized cardiolipin, and thus the green fluorescence was reduced. Accordingly, the relative fluorescence intensity was recorded to quantify cardiolipin oxidation. MitoQ was added to the medium of PANC-1 cells to neutralize the mROS that were produced by mitochondrial fragmentation. **i** mPTP opening was determined using tetramethylrhodamine ethyl ester. The relative mPTP opening rate was quantified as a ratio to that of control group. *p < 0.05

At the molecular level, HtrA2/Omi is primarily expressed in the inner membrane of mitochondria. Based on a recent study, the liberation of HtrA2/Omi from mitochondria into the cytoplasm is dependent on cardiolipin oxidation and mPTP opening [15, 44]. First, the oxidation of cardiolipin lowers the affinity of HtrA2/Omi to the mitochondria. Second, the opening of mPTP provides a channel for HtrA2/Omi leakage [45]. Given the role of mitochondrial fragmentation in cellular oxidative stress via mROS overproduction, we asked whether mROS was required for the mitochondrial fragmentation-mediated HtrA2/Omi liberation via modulating cardiolipin oxidation and mPTP opening. To support our hypothesis, cardiolipin oxidation was determined via staining with NAO, which is a cardiolipin probe. Under physiological conditions, NAO could interact with cardiolipin to display a green fluorescence. In response to cardiolipin oxidation, NAO cannot bind to oxidized cardiolipin, and thus the green fluorescence is reduced. As shown in Fig. 4g, h, the fluorescence of cardiolipin was significantly downregulated in response to erlotinib, and this effect was reversed by Mdivi-1. To verify whether mROS was responsible for cardiolipin oxidation, mitoQ was used to neutralize the mitochondrial fragmentation-produced mROS. Interestingly, mitoQ treatment also reversed the green fluorescence intensity of cardiolipin (Fig. 4g, h), similar to the results obtained via supplementation with Mdivi-1. These results verified the role played by mROS in cardiolipin oxidation. In addition, we also found that the mPTP opening rate was significantly increased in response to erlotinib (Fig. 4i), and this effect was inhibited by Mdivi-1 or mitoQ (Fig. 4i). Together, our data demonstrated that the mitochondrial fragmentation-mediated mROS regulated HtrA2/Omi liberation via inducing cardiolipin oxidation and mPTP opening.

RETRACTED

### Released HtrA2/Omi induces caspase-9-dependent apoptosis

After it is released into the cytoplasm, HtrA2/Omi can interact with and activate mitochondrial apoptosis in a manner that is dependent on caspase-9 activity [11]. Notably, an early feature of caspase-9-related apoptosis is the reduction of mitochondrial potential. In the present study, a JC-1 kit was used to stain for the mitochondrial potential. The results indicated that erlotinib treatment significantly reduced the mitochondrial potential (Fig. 5a, b), and this effect was inhibited by Mdivi-1. To confirm whether HtrA2/Omi accounted for the mitochondrial potential collapse, two independent siRNAs were used. After knockdown of HtrA2/Omi, the mitochondrial potential was analyzed again. Compared to the erlotinib-treated group, the loss of HtrA2/Omi stabilized the mitochondrial potential (Fig. 5a, b), an effect that was similar to the results obtained via treatment with Mdivi-1. Furthermore, the last characteristic of caspase-9-related apoptosis is the activation of caspase-9, an effect that is accompanied by an increase in proapoptotic proteins. In the present study, the protein activity (Fig. 5c) and expression (Fig. 5d, e) of caspase-9 were both upregulated in answer to erlotinib stress and these effects could be repressed by Mdivi-1 or HtrA2/Omi siRNA. As a consequence of caspase-9 activation, the levels of proapoptotic factors such as Bad and Bax were significantly increased in response to erlotinib treatment, and this effect was negated by Mdivi-1 treatment or HtrA2/Omi siRNA transfection (Fig. 5f–j). By comparison, the expression of antiapoptotic proteins, including Bcl-2 and survivin, were obviously downregulated by erlotinib (Fig. 5f–j) and were reversed to near-normal levels with Mdivi-1 treatment or HtrA2/Omi knockdown. Together, our results indicated that mitochondrial fragmentation activated caspase-9-dependent apoptosis via HtrA2/Omi.

**Fig. 5:** Released HtrA2/Omi triggers an activation of caspase-9-related cellular apoptosis. **a**, **b** The mitochondrial potential was determined using a JC-1 kit in PANC-1 cells. Mdivi-1 was used to inhibit mitochondrial fragmentation. Furthermore, two independent siRNAs against HtrA2/Omi were transfected into PANC-1 cells to suppress HtrA2/Omi expression. The red-to-green ratio was recorded to quantify the mitochondrial potential. **c** The activation of caspase-9 was measured using an ELISA to evaluate the activity of caspase-9. Mdivi-1 was used to inhibit mitochondrial fragmentation. Furthermore, two independent siRNAs against HtrA2/Omi were transfected into PANC-1 cells to suppress HtrA2/Omi expression. **d**, **e** Expression of caspase-9 was determined via immunofluorescence. **f**–**j** Western blotting was performed to detect alterations in proapoptotic proteins and antiapoptotic factors. Mdivi-1 was used to inhibit mitochondrial fragmentation. Additionally, two siRNAs against HtrA2/Omi were transfected into PANC-1 cells to suppress HtrA2/Omi expression. *p < 0.05

### Mitochondrial fragmentation also modulated PANC-1 cell proliferation via mROS-HtrA2/Omi pathways

To this end, we asked whether mitochondrial fragmentation was involved in PANC-1 cell proliferation via the mROS-HtrA2/Omi pathways. First, the EdU assay was conducted to observe cellular proliferation. As shown in Fig. 6a, b, compared to the control group, erlotinib treatment significantly reduced the ratio of EdU-positive cells; this effect was repressed by Mdivi-1 (Fig. 6a, b). In addition, the neutralization of mROS via mitoQ and knockdown of HtrA2/Omi via siRNA transfection also reversed the number of EdU-positive cells after erlotinib treatment (Fig. 6a, b). These results indicated that mitochondrial fragmentation affected the cell proliferation in PANC-1 cell via the mROS-HtrA2/Omi axis. Further, the cell proliferation is primarily regulated by CDK4 and Cyclin D1. Cyclin D1 and cyclin E interact with each other and generate cyclin-dependent kinase (Cdk)4/6-cyclin D and/or Cdk2-cyclin E complexes, which accelerate transition from the G0/G1 to S stage, according to the previous study [46]. We have provided the references for this. With the help of a western blotting assay, we found that the expression of CDK4 and Cyclin D1 were both reduced in response to erlotinib treatment, and this effect was negated by Mdivi-1 (Fig. 6c–e). Interestingly, the neutralization of mROS via mitoQ and knockdown of HtrA2/Omi via siRNA transfection also reversed the levels of CDK4 and Cyclin D1. Together, our results confirmed that PANC-1 cell proliferation was modulated by erlotinib via mitochondrial fragmentation in a manner that was dependent on the mROS-HtrA2/Omi pathways.

RETRACTED

**Fig. 6:** Mitochondrial fragmentation regulates the proliferation of PANC-1 cells via the mROS-HtrA2/Omi pathways. **a** The EdU assay was used to observe the cellular proliferation in response to erlotinib treatment. Mdivi-1 was used to inhibit mitochondrial fragmentation. Furthermore, two siRNAs against HtrA2/Omi were transfected into PANC-1 cells to suppress HtrA2/Omi expression. Additionally, mitoQ was added into the medium of PANC-1 cells to attenuate the production of mROS. **b** The quantification of EdU-positive cells. **c**–**e** CDK4 and Cyclin D1 expression were evaluated via western blotting. Mdivi-1 was used to inhibit mitochondrial fragmentation. In addition, two siRNAs against HtrA2/Omi were transfected into PANC-1 cells to suppress HtrA2/Omi expression. Furthermore, mitoQ was added to the medium of PANC-1 cells to attenuate the production of mROS. *p < 0.05

## Discussion

According to the previous findings, mitochondrial fission has been acknowledged as a potential target to reduce the proliferation, migration and survival of PANC-1 pancreatic cancer cells [10]. Excessive mitochondrial fission promotes mitochondrial fragmentation [15]. Fragmented mitochondria induce damage to mitochondrial structure and function, eventually interrupting the cellular ATP supply and activating the apoptosis response [47, 48]. However, the detailed molecular mechanism by which mitochondrial fragmentation triggers mitochondrial damage and cellular apoptosis remains unclear. Our study provides an answer to this question. We used different doses of ERL to screen its proapoptotic effect in two types of cancer cell lines. Then, we used the minimal lethal dose of ERL to investigate its apoptotic mechanism, with a focus on mitochondrial damage. We observed the minimal lethal dose of ERL has an ability to induce the mitochondrial fragmentation and this finding may explain one of the mechanisms by which ERL mediated cancer cell apoptosis. Notably, whether higher dose of ERL could activate other signaling pathway to induce cell apoptosis requires further investigation. Our data illustrated that erlotinib treatment promoted mitochondrial fragmentation that occurred via increased mitochondrial fission and decreased mitochondrial fusion. Subsequently, excessive mitochondrial fragmentation triggered mROS overloading, leading to cellular oxidative stress and disordered energy metabolism. In addition, mROS overproduction was closely associated with cardiolipin oxidation and mPTP opening, favoring HtrA2/Omi liberation from mitochondria into the cytoplasm. As a consequence of HtrA2/Omi leakage, reduction of the mitochondrial potential and caspase-9 activation were noted, and these alterations were accompanied by an upregulation of proapoptotic proteins and a downregulation of antiapoptotic factors. Overall, we demonstrated for the first time that erlotinib-activated mitochondrial fragmentation mediated PANC-1 apoptosis via the mROS-HtrA2/Omi pathways. This finding fills the knowledge gap regarding how mitochondrial fragmentation induces mitochondrial damage and triggers the apoptotic pathway.

RETRACTED

Mitochondrial fission and fusion are a part of mitochondrial dynamics. Under physiological conditions, the mitochondrial network undergoes moderate fission and fusion to fill the requirements for cellular metabolism [49, 50]. Mild levels of mitochondrial fission help the mitochondria in generating daughter mitochondria, whereas moderate levels of mitochondrial fusion provides the energy for communication between the mitochondrial network [51, 52]. Interestingly, uncontrolled mitochondrial fission generates massive amounts of fragmented mitochondria and disrupts mitochondrial homeostasis. Previous studies have identified mitochondrial fragmentation, which is produced by mitochondrial fission, as the apoptotic trigger in various disease models. For instance, in fatty liver disease, mitochondrial fragmentation promotes the apoptosis of hepatocytes and the progression of liver fibrosis by decreasing mitophagy [53]. In neurodegenerative illness such as Alzheimer’s disease, excessive mitochondrial fragmentation disturbs mitochondrial energy metabolism and causes neuronal oxidative injury [54]. In addition, in rectal cancer, activated mitochondrial fragmentation limits tumor proliferation and augments cancer apoptosis [11]. In accordance with these findings, our data also illustrated the necessary role played by mitochondrial fragmentation in initiating pancreatic cancer PANC-1 cell death. Thus, mitochondrial fragmentation would be considered as a tumor-suppressor, and strategies to promote mitochondrial fragmentation are of significant importance in the design of anti-cancer drugs.

Although the proapoptotic effect of mitochondrial fragmentation has been well-documented, the detailed mechanisms by which mitochondrial fragmentation induces mitochondrial damage and activates cellular apoptosis are incompletely understood. In the present study, we found that mitochondrial fragmentation modulated mitochondrial homeostasis and cell viability through two mechanisms. One mechanism was driven by the promotion of mROS-mediated cell oxidative injury, and the other involved the HtrA2/Omi liberation-induced caspase-9 activation. First, mitochondrial fragmentation generated superfluous amounts of mROS, and the excess mROS induced cardiolipin oxidation and mPTP opening [55]. Subsequently, oxidized cardiolipin and increased mPTP opening worked together to augment the liberation of HtrA2/Omi from mitochondria into the cytoplasm, where Htra2/Omi reduced the mitochondrial potential and induced caspase-9 activation. This information was also consistent with previous studies. In cardiac ischemia–reperfusion injury, excessive mitochondrial fragmentation-induced mitochondrial DNA damage evokes mROS overproduction and cardiolipin oxidation [14, 15]. Additionally, in oral cancer, mitochondrial fragmentation-related cardiolipin oxidation and mPTP opening eventually contribute to caspase-involved cellular apoptosis [56].

In the present study, we used erlotinib to activate mitochondrial fragmentation and found that erlotinib-mediated PANC-1 cellular apoptosis could be inhibited by Mdivi-1, which is an antagonist of mitochondrial fragmentation. To the best of our knowledge, this is the first study to investigate the role of erlotinib in mitochondrial stress. Although erlotinib has been tested in several human clinical studies [57, 58], its pharmacological mechanism has not been adequately explored. Our study proposed that the anti-cancer property of erlotinib relied on the activation of mitochondrial fragmentation by upregulating mitochondrial fission and downregulating mitochondrial fusion. Notably, the dose selection of ERL was according to a previous study [26] and this selection may be also relied on the types of cancer cell lines. In clinical practice, different doses of ERL have been used according to the tumor staging and pathologic grading. Further insight is required to figure out the appropriate concentration of ERL on different types of pancreatic cancer. Besides, there are several limitations in the present study. Although we used two pancreatic cancer cell lines to screen the role of erlotinib, an animal study is necessary to further support our finding. In addition, human evidence is also required to validate the tumor-suppressive effects of mitochondrial fragmentation in response to erlotinib treatment.

RETRACTED

## Conclusion

Collectively, our results reported that mitochondrial fragmentation, which was activated by erlotinib, regulated the viability of the PANC-1 pancreatic cancer cell line via the mROS-HtrA2/Omi pathways. This conclusion provides a potential target to modify pancreatic cancer viability via augmenting mitochondrial fragmentation and activating the mROS-HtrA2/Omi pathways.

## Additional file

**Additional file 1: Figure S1.** The proapoptotic effect of erlotinib on PANC1 cells using Annexin V/PI staining. Early apoptosis (Annexin V+/PI- cells) and late apoptosis (Annexin V+/PI+ cells) were counted. #*p*<0.05 *vs.* control group.
